# Wearable Running Training Data Acquisition System Based on Intelligent Computer Technology

**DOI:** 10.1155/2022/4508570

**Published:** 2022-07-01

**Authors:** Ruirui Zhang, Zhao Liu, Zhansheng Chang, Yongqing Cao, Dan Liu

**Affiliations:** School of Computer Science and Engineering, Cangzhou Normal University, Cangzhou 061001, China

## Abstract

Because the instantaneous motion of running training changes rapidly, the acquisition accuracy is low. Therefore, a wearable running training data acquisition system based on intelligent computer technology is designed. In the hardware design of the system, by setting the registers of the main control chip, inertial sensor, and magnetic sensor, the acceleration and angular velocity information of motion exist in the data format of binary complement. Bluetooth realizes the transparent transmission of data between hardware and software. The system software uses LDA recognition algorithm to decompose the dynamic data transmitted by Bluetooth into multiple static data and collect the final motion data through training. The experimental results show that the designed system has good quality and high accuracy in motion detection and counting.

## 1. Introduction

In recent years, with the rapid improvement of living standards, people began to pay more and more attention to health issues, coupled with the improvement of urban sports facilities and the strong call of the state for national fitness. More and more people begin to form the habit of exercise and running. Sports and fitness have gradually become a part of people's life [1–3]. However, compared with people's growing enthusiasm for sports, the growth of sports software and hardware seems to lag behind. Because there is no corresponding equipment to record their own movement, the movement record will be lost over a long time, so people cannot better plan their own movement plan [4]. In addition, most people lack enough sports knowledge and do not know how to exercise properly and with high quality. Excessive and incorrect sports will burden the body of athletes and even cause permanent damage. However, professional gyms or fitness coaches need to spend a lot of money and are inconvenient. It is obviously not a good choice for students, ordinary white-collar workers, and other gyms. These problems lead to boredom in the exercise process and unsatisfactory exercise effect [5]. However, with the rapid development of smart phones and mobile networks, and the emergence and popularization of wearable devices such as various sports bracelets, sports records are more accurate and comprehensive. A large number of sports online tutorials can also make it easier and faster for people to obtain all kinds of sports knowledge and even obtain special sports plans based on their own sports status [6–9]. These advantages make the combination of IT and sports more and more popular. Various companies have also launched a variety of sports APP and launched free sports records, fitness guidance, and other services to attract users and seize this emerging market [10, 11]. In addition to sports itself, the concept of sports social networking is becoming more and more mature and loved by users and has even become a keyword that sports APP need to pay attention to. Sports social networking is a new social model based on sports. Due to the rise of online social networking and the continuous encouragement and support of the state for sports, sports social networking is for young people, it has become a new way to communicate with friends [12–14]. Sports social networking meets the social needs of modern young people and brings stable user traffic and large user stickiness to sports APP. Therefore, these sports APP can also refer to some current social media, such as microblog and WeChat, so as to bring formal profits to the emerging market of sports [15–17].

This paper proposes a wearable running training data acquisition system based on intelligent computer technology. Intelligent computer technology refers to a new computer technology that can simulate, extend, and expand human intelligence. It can store a large amount of information and knowledge, can reason, deduce, and summarize, has learning function, and can use natural language, text, sound, and graphics. The structure of exchanging information and knowledge between images and people is a general-purpose high-speed parallel processing computer. It is an organic combination of modern computing technology, communication technology, and artificial intelligence and bionics and provides a tool for knowledge processing. Based on the in-depth research on bracelets, watches, wearable devices, and existing sports software, a targeted and attractive sports software scheme is proposed. Technically speaking, considering the convenience and high popularity of the current development of computer technology, the innovation of the research content has carried out the exploration of related sensors in combination with motion technology and plans to develop other related motion sensors when the types of sensors increase in the future.

## 2. Hardware Environment Design Based on CCS

In fact, intelligent computer technology has become a dynamic development concept, which is always at the forefront of computer technology. The task of artificial intelligence is to study unsolved computer problems, which reflects the remarkable characteristics of artificial intelligence and intelligent computer research different from other disciplines. Intelligent application problems often adopt the search method without a definite solution algorithm. Once people have mastered enough knowledge of a problem, that is, they have found a definite algorithm that does not need search, and their behavior and effect can be predicted, this problem is generally no longer regarded as an intelligent problem. At present, knowledge base, which is regarded as the main part of intelligent computer, will be regarded as general intelligent computer technology like database in the near future. Therefore, intelligent computer is regarded as a high technology that drives the continuous development of computer rather than a machine completely different from traditional computer. This pressure forces researchers engaged in intelligent computer research to constantly put forward new concepts and methods and constantly overcome new technical difficulties. The running training data acquisition system designed in this paper is realized by establishing nonhierarchical acquisition nodes at the acquisition end and configuring the child nodes and parent nodes accordingly [18, 19]. The child node is responsible for data collection and the parent node is responsible for data summary. The acceleration and angular velocity sensors and magnetic sensors used at the data acquisition end are digital sensors. Therefore, in addition to the configuration of the main control chip, the sensors also need to be configured [20–22]. When initializing and configuring MPU6050, HMC5883, and CS5509 chips and reading data, it is necessary to write and read registers through I2C bus [23–25]. The process of I2C bus register writing is generally as follows: the main device sends the start signal. The master device sends the I2C address (7 bits) and write operation bit 0 (1 bit) of the slave device, waiting for the response signal, and sends a response signal from the device. The main device sends the register address (8 bits) and waits for the response signal and sends a response signal from the device. The main device sends the data to be written into the register (8 bits) and waits for the response signal and sends a response signal from the device (the above two steps can be repeated many times to write multiple register data). The main device sends a stop signal. The process of I2C bus register reading is as follows: the main device sends the start signal. The master device sends the I2C address (7 bits) and write operation bit 0 (1 bit) of the slave device, waiting for the response signal, and sends a response signal from the device. The main device sends the register address (8 bits) and waits for the response signal and sends a response signal from the device. The main device sends the start signal. The master device sends the I2C address (7 bits) and read operation bit 1 (1 bit) of the slave device, waiting for the response signal, sends a response signal from the device, and sends data from the device register (8 bits). After the main device reads the data and sends a response signal, it sequentially reads multiple register data. The main device sends a nonresponse signal. The main device sends a stop signal. The configuration of this paper is to set the register directly. The specific design is as follows.

### 2.1. Configuration of Main Control Chip MSP430G2553

Power on initialization, basic clock system configuration, general I/O port configuration, timer configuration, serial port configuration and ADC (Analog-to-Digital Converter) configuration. Details are as follows:

1. Basic clock system configuration: MSP430g2553 has a rich clock system to support very low system consumption. It has three clock sources: standard 32.768 kHz external clock source (LFXT1CLK), low frequency and low power 12 kHz internal clock source (VLOCLK), and internal programmable digital clock source (DCOCLK). At the same time, three clock signals are provided, including peripheral auxiliary clock (ACLK), master clock (MCLK), and secondary clock (SMCLK). The configuration sequence is as follows: configure the clock source, configure the main clock and secondary clock frequency divider, write the adjustment value according to the required digital clock, and configure the peripheral clock frequency divider
2. General I/O port configuration: the interfaces used include power monitoring (P1.0), red indicator (P1.3), green indicator (P1.4), wireless module setting (P1.5), I2C clock line (P2.0), I2C data line (P2.1), magnetic sensor interrupt (P2.2), and inertial sensor interrupt (P2.5). Configure interface function and interface direction, enable resistance, clear flag bit, interrupt enable, and trigger mode
3. Timer configuration: select timer 0 as sampling timer and timer 1 as timeout timer. The configuration sequence is as follows: set the time, select the clock source and frequency divider, count mode, timer reset, trigger mode, enable interrupt, and timer 1 has high priority
4. Serial port configuration: select clock source, set baud rate, configure interface function, clear flag bit, and receive interrupt enable
5. ADC configuration: use ADC to monitor the battery power supply, 10 bit analog-to-digital converter, the maximum conversion rate is 200 ksps, and has 8-channel external input. The configuration sequence is as follows: clear flag bit, interrupt enable, reference voltage selection, turn on internal reference voltage, select sampling rate and holding time, select sampling mode, select input channel, and select clock source and frequency divider. ADC configuration is used to convert analog signals with continuous time and continuous amplitude into digital signals with discrete time and discrete amplitude. Generally, it goes through four processes: sampling, holding, quantization, and coding. In the actual circuit, some of these processes are combined. Sampling and holding, quantization, and coding are often realized simultaneously in the conversion process, which has high resolution and can reduce the conversion error

### 2.2. Configuration of Inertial Sensor MPU6050

The important registers of MPU6050 are shown in Table 1.

The initialization configuration of MPU6050 is as follows: selection of internal 8 M clock source, configuration of sampling rate, configuration of acceleration angular velocity low-pass filter and range selection, and data preparation interrupt enable. The data format stored in the acceleration and angular velocity register is binary complement, and the conversion formula of acceleration and angular velocity is

(1) $$\begin{array}{c} A_{\text{accelData}}=\frac{R_{\text{registerAccel}}}{A_{\text{AccelSensitivity}}},\\ G_{\text{gyroData}}=\frac{R_{\text{registerGyro}}}{G_{\text{GyroSensitivity}}}. \end{array}$$

Among them, *A*_accelData_ represents acceleration data, *R*_registerAccel_ represents running speed result, *A*_AccelSensitivity_ represents running speed change sensitivity, *G*_gyroData_ represents rotation data, *R*_registerGyro_ represents running angular speed result, and *G*_GyroSensitivity_ represents running angular speed change sensitivity.

Because the action data requires high real-time performance, in the processing of inertial data, in addition to threshold filtering and selecting the range according to the actual situation, the high sampling rate of the sensor is also used for average filtering.

### 2.3. Configuration of Magnetic Sensor HMC5883

Magnetic sensor HMC5883 is the key part of data acquisition. The performance of magnetic sensor determines the accuracy of data acquisition system. The important registers of HMC5883 are shown in Table 2.

The initialization configuration of HMC5883 is as follows: sampling rate configuration, 8 sampling data for one measurement data output, output rate configuration of 30 Hz, measurement mode configuration, and range selection. The storage format of magnetic field data in the register is binary complement, and the conversion formula of magnetic field intensity is

(2) $$\begin{array}{c} M_{\text{magData}}=\frac{R_{\text{registerMag}}}{G_{\text{Gain}}}, \end{array}$$

where *M*_magData_ represents the magnetic field strength data,  *R*_registerMag_ represents the actual result of the magnetic field, and *G*_Gain_ represents the binary complement.

The processing of magnetic field data is the same as that of inertial data. The appropriate range and threshold filtering are selected, and the data average filtering is carried out by using the register of the sensor itself.

## 3. Software Environment Design

### 3.1. Transparent Transmission of Collected Data

The serial port connection of wearable devices is the basis of real-time data transmission, so it also communicates through serial port. This paper takes Bluetooth as the connection mode, and the data transmission process of Bluetooth transparent transmission module is shown in Figure 1.

As can be seen from Figure 1, according to the data transmission process based on Bluetooth technology, the Bluetooth transparent transmission module of wearable device is designed. The HC-05 Bluetooth serial communication module designed in this paper is a widely used Bluetooth transparent module. Transparent transmission is the simplest communication mode in Bluetooth transmission. In the transmission, there is no need to process the data according to the transmission protocol. Like wired serial port, it can directly send the data through Bluetooth. The transparent transmission module enables developers to quickly realize the data transmission function based on Bluetooth without learning the underlying protocol of Bluetooth. The module is 27 mm long, 13 mm wide, 2 mm thick, compact, and easy to integrate into the system. The module can realize Bluetooth transmission within 10 m. The working power supply voltage is 3.3 V. It is connected with the serial port of Arduino through the serial port. Improve the convenience of wearing. When HC-05 receives the command data from the mobile phone, it sends it to Arduino due through the serial port. When Arduino due reads the command to send sensor data, it transmits the data to the Bluetooth transparent module HC-05 through the serial port and then sends it to the mobile phone. Bluetooth transparent module HC-05 plays a bridge role in wireless data transmission.

### 3.2. Running Motion Recognition Based on LDA Recognition Algorithm

When analyzing the data transmitted through Bluetooth, the movement exists in dynamic mode in the process of running training. A dynamic action mode can be decomposed into many static action modes; that is, the collected signals of dynamic action modes actually correspond to countless different static action modes, which makes the dynamic action mode more complex and difficult to identify than the static action mode. The calculation process of LDA Algorithm is simple and suitable for transplanting the recognition program to wearable devices. However, for the dynamic action mode of lower limbs, the pattern recognition algorithm for static action mode cannot be directly applied, so it is necessary to identify the dynamic action mode through another method. In order to recognize dynamic action patterns, a pattern recognition algorithm based on phase interception is used in this paper. The dynamic movement mode of running is that the lower limbs repeatedly complete an action cycle, and the action cycles of these actions can be described as a gait macroscopically. Taking the right foot as the research object, each gait starts from the rear heel landing of the right foot to the next rear heel landing of the right foot. For the static action mode, the value of the signal is often stable, so that the data can be divided into windows. The data of each data window after segmentation has a high degree of unity. The gait of dynamic action mode has a relatively large action amplitude; that is to say, all kinds of signals of each gait change greatly, so the data window cannot be segmented directly as for static action mode.

Although the various signals of the dynamic action mode are constantly changing, each gait cycle has the time nodes of heel touchdown and forefoot touchdown. According to the numerical change trend of the plantar pressure sensor of the experimental system, the time points of heel touchdown and forefoot touchdown of each gait can be detected. The relationship between plantar pressure and time can be expressed as

(3) $$\begin{array}{c} P=\left(mg+F\right)\left(\frac{\left|t-t_{\text{mid}}\right|}{T}\right), \end{array}$$

where *P* represents the plantar pressure value, *m* represents the weight of the runner, *g* represents the gravity coefficient, *t*_mid_ represents the middle time of completing a running action, *t* represents the acquisition time, and *T* represents the time of completing a running action.

On this basis, if a small segment of sensor data is intercepted near a fixed time point, the data will be relatively stable because of the short time, and the data of the same stage can be intercepted in each gait, so that the data of different data windows have good unity. The static pressure value *p* at this time can be expressed as

(4) $$\begin{array}{c} p=\left(\frac{\min\left|t-t_{\text{mid}}\right|}{T}\right)\left(mg+F\right), \end{array}$$

where min|*t* − *t*_mid_| represents the minimum time period length of interception.

At this time, the data window intercepted at the fixed stage of each gait according to the plantar pressure can be used to distinguish different dynamic action modes after being processed by the pattern recognition algorithm.

This paper intercepts the data of the fixed stage of gait based on plantar pressure. There is a complete gait process between two heel touches of the same foot. For the pressure signals of the rear heel and front sole, when the signal is greater than the threshold, it means touching the ground, and when the signal is less than the threshold, it means hanging off the ground. In the actual running training process, the pressure value of the rear heel increases above the threshold before the pressure value of the front sole and decreases below the threshold before the pressure value of the rear heel. For the whole time from the heel landing to the forefoot landing, the foot does not leave the ground, so it is called the standing phase, and other times in the gait are called the swing phase. The pressure change function at this time is

(5) $$\begin{array}{c} f\left(t\right)=p\left(\frac{\left|t-t_{\text{mid}}\right|}{T}\right), \end{array}$$

where *f* is the pressure variation function.

Since there must be two key nodes in each gait cycle (rear heel touchdown and front foot off the ground), based on this, the sensor data of *T* period before and after rear heel touchdown and *t* period before and after front foot off the ground in the gait cycle are intercepted according to the pressure information of plantar sensor, and the detailed definitions and abbreviations of these four stages are shown in Table 3.

According to Table 3, a gait cycle of running dynamic action mode is intercepted at four different stages. In pattern recognition, it is necessary to select one of the four stages as the data window and then select the data of this stage for recognition. Because the length of the stage is *t* period, the data of the stage can be directly used as the data window. The data window is used for feature extraction, and the five primary time-domain features of absolute mean, variance, root mean square, and Wilson amplitude are calculated for later training and recognition. After selecting the optimal feature combination, half of the feature vectors belonging to different action modes are trained, half of them are recognized, and the recognition rate is counted. The training method is

(6) $$\begin{array}{c} D=\lambda \left(\bar{f\left(t\right)}+\varepsilon +\kappa +\gamma \right), \end{array}$$

where *D* represents the training result, *λ* represents the training coefficient, $\bar{f\left(t\right)}$ represents the absolute mean value of the data, *ε* represents the variance of the data, *κ* represents the root mean square of the data, and *γ* represents the amplitude of the data.

After intercepting the signal of dynamic action mode and obtaining the feature vector, in the training process, for different dynamic action modes, the feature vector extracted from the data in the same stage is trained with LDA algorithm to obtain the dimension reduction matrix and the label vector of each dynamic action mode. In the process of recognition, the dimension of the intercepted feature vector is reduced by the dimension reduction matrix, and then, the recognition result is obtained by comparing the Euclidean distance between the reduced feature vector and the label vector. The calculation method is

(7) $$\begin{array}{c} f\left(t\right)=\frac{\left(d+b\right)}{l}, \end{array}$$

where *d* represents the feature vector, *b* represents the label vector, and *l* represents the Euclidean distance.

## 4. Dynamic Test

In order to verify the overall effectiveness of the wearable running training data acquisition system based on intelligent computer technology, this method needs to be tested. The CPU used is Pentium (R) dual core, the system is Windows 7, the processor is core i5, the main frequency is 2.5 GHz, the platform is MATLAB, the memory is 8 GB, and the hard disk is 120 g. The simulation experiment of the steady-state training method of the software is carried out.

### 4.1. Test Condition Setting

Taking daily running behavior as an example, multisensor data acquisition terminal is used to collect limb movement data. The first group of actions selects the repetitive process from standing upright to completing a run, repeats the above actions for 35S, and counts the collection results. Both running and standing are relatively static posture, and the leg posture can accurately reflect the human action. The data acquisition end is installed on the side of the right leg, and the wearing effect is shown in Figure 2.

### 4.2. Test Results

Based on the above, this paper compares the data information of actual running with the data collected by the system, and the results are shown in Figure 2.

As can be seen from Figure 3(a), the acceleration acquisition results of the system designed in this paper have a high degree of fit with the actual results and can realize accurate control for the changed nodes. There are 5 acceleration changes in the running process, and the time error acquisition results of the system are no more than 0.1 M. By observing Figure 3(b), it can be seen that the system also has high accuracy in the collection of running angular velocity change data. In the whole experimental process, although the change range of angular velocity is within 5°, the system still realizes the effective collection of angular velocity. It shows that the system designed in this paper can effectively collect running training data.

To sum up, the wearable running training data acquisition system based on intelligent computer technology has high accuracy in the collection of running acceleration and angular velocity change data and can effectively collect running training data.

## 5. Conclusion

With people's attention to sports, sports software will have better market demand. A good sports software should not only have the most basic sports data recording function. Based on the data, this topic attempts to provide cheap and reliable exercise guidance by using ready-made mobile phones and sensors and tries to develop an integrated health exercise system by using different types of sensors and the concept of plug-in development. By collecting, analyzing, and processing the data of mobile phone sensors, generate corresponding motion data, analyze according to the relevant data, recommend reasonable motion plans for users, provide standardized sports teaching of corresponding projects, make statistical analysis, and display and share the motion situation. Through the above functions, users can use the system for a long time and produce user stickiness. After sufficient market demand research and relevant technology research, the system development is completed based on Android+Java technology. The main research results are as follows:

1. Starting with the background research and the practical application of the system, based on the existing shortcomings of similar products, the analysis of the application of sensor data into different types of motion and the data used in the development process
2. The algorithm of human motion information acquisition system and the design of each functional module and database design
3. The system is implemented based on Android and Java technology, and the system functions and performance tests are completed. The test results show that the system has good quality, and the motion detection and counting also achieve high accuracy

The research on the design and implementation of sports information acquisition system has effectively developed an integrated music power system about healthy sports. However, there are still some deficiencies that need to be continuously improved. Due to limited time, only basic functions have been completed, and more functions to attract users need to be further added. The following aspects can be studied in the future:

1. Further improve the LDA recognition algorithm to minimize the error. Design the wireless transmission module to achieve longer transmission distance and less power consumption. Enrich the functions of the wearable running training data acquisition system and analyze the real-time data of running training as much as possible to achieve better results
2. Integrate other physical training items into the system, such as push ups, sit ups, squats, and pull ups. Judge whether each item reaches the qualified level by monitoring the changes of trainees' joints or the changes of relative positions between their bodies
3. More information collection modules are introduced and distributed in various locations of running training clothes, and the collected information (positioning information, physiological data information, etc.) is integrated and applied to the future highly information-based market competition

## Figures and Tables

**Figure 1:** Data transmission process based on Bluetooth.

**Figure 2:** System wearing effect.

**Figure 3:** Running data collection results. (a) Acceleration data acquisition results. (b) Angular velocity acquisition results.

**Table 1:** Register configuration of MPU6050.

Register name	Register address	Explain
SLAVEADDRESS1	0xd0	Register operation address
SMPLRT_DIV	0x19	Sample rate divider
PWR_MGMT	0x6b	Power management and clock configuration
CONFIG	0x1a	Low pass filter configuration
GYRO_CONFIG	0x1b	Gyroscope self-test and range selection
ACCEL_GONFIG	0x1c	Angular velocity data register group
INT_ENABLE	0x38	Interrupt configuration
GYRO_OUT	0x43~0x48	Angular velocity data register group
ACCEL_OUT	0x3b~0x40	Acceleration data register group

**Table 2:** Register configuration of HMC5883.

Register name	Register address	Explain
SLAVEADDRESS2	0x3c	Register operation address
CONFIG_A	0x00	Selection of sampling times and output rate
CONFIG_B	0x01	Range selection
MODE	0x02	Measurement mode selection
DATA_X	0x03 0x04	X
DATA_Y	0x07 0x08	Y
DATA_Z	0x05 0x09	Z
STATUS	0x09	Data register status monitoring

**Table 3:** Definitions and abbreviations of four stages.

Serial number	Name	Abbreviation	Detailed definition
1	Pretouchdown stage of rear heel	Pre-FC	*t* period before heel touchdown
2	Postheel touchdown stage	Post-FC	*t* period after heel touchdown
3	Pretouchdown stage of rear forefoot	Pre-FO	*t* period before forefoot touchdown
4	Postforefoot touchdown stage	Post-FO	*t* period after forefoot touchdown

## Data Availability

The data used to support the findings of this study are available from the corresponding author upon request.
